# Weight status of adolescents in secondary schools in port Harcourt using Body Mass Index (BMI)

**DOI:** 10.1186/1824-7288-38-31

**Published:** 2012-07-23

**Authors:** Adesuwa F Adesina, Oliemen Peterside, Ifeoma Anochie, Nwadiuto A Akani

**Affiliations:** 1 Department of Paediatrics, Randle General Hospital, Surulere, Lagos State, Nigeria; 2 Department of Paediatrics and Child Health, Niger Delta University Teaching Hospital, Okolobiri, Bayelsa State, Nigeria; 3 Department of Paediatrics, University of Port Harcourt Teaching Hospital, Alakahia, Port Harcourt, Nigeria

**Keywords:** Adolescents, Weight status, Body mass index

## Abstract

**Background:**

Adolescent weight status is a cumulative effect of health and nutritional problems. Adolescent weight problems often go unnoticed as weight assessment is not considered a priority in adolescents.

**Objectives:**

To determine the weight status of adolescents using BMI and to identify the contributing factors to adolescent weight problems.

**Methods:**

In April 2010, 960 adolescents aged 10–19 years in secondary schools in Port Harcourt were selected for the study using a stratified multi-staged sampling method. Structured questionnaires were filled by the investigators while weight and height were measured. BMI was calculated using the formula weight/height^2^ (kg/m^2^).

**Results:**

The prevalence of underweight, overweight, obesity and stunting were 6.4%, 6.3%, 1.8% and 5.4% respectively. Factors which were commoner in overweight adolescents were high socioeconomic class, higher maternal education, spending > 3 hours a day watching television and frequent ingestion of snacks.

**Conclusion:**

There is a need for periodic weight assessment of adolescents and health education to promote healthy eating habits and regular physical exercise as part of the School Health Programme.

## Introduction

Adolescence refers to the developmental period between childhood and adulthood. The World health organization (WHO) defines adolescents as individuals between the ages of 10–19 years and they make up about 20% of the world’s population [1,2]. There are about 1.2 billion adolescents in the developing nations, making up one fifth to one quarter of the population [3].

Adolescence is the second most critical period of physical growth after the first year [4,5]. It is a time of enormous physiological, cognitive and psychosocial changes, largely dependent on hormonal and environmental influences [4,6]. Twenty five percent of adult height, and up to fifty percent of adult weight are attained during adolescence [4,7]. It is also a time of sexual development and increase in fat especially in girls and muscle mass in boys [8]. The demands of this normal physical growth and maturation lead to increased need for nutrients and micronutrients like vitamins A, B_12_, C, folic acid, calcium and iron. This places extra nutritional demands on adolescents [8]. A combination of the energy demands of the adolescent growth spurt and inadequate diet has contributed a lot to the poor weight status of adolescents.

Adolescent weight status is a cumulative effect of the health and nutritional problems occurring during early childhood as well as those originating in adolescence. Previous studies have shown that adolescents suffer from a range of health problems especially those associated with substance abuse, sexual behaviour and poor eating habits [9]. For many of them, inadequacies of the quality and quantity of food they eat, are the prime causes of weight problems which often go unnoticed since assessment of weight status is not considered a priority in adolescence as it is in children [9,10].

Although, studies on adolescent weight status have focused on undernutrition, some adolescents have the problem of overnutrition (obesity) [9,11-15]. Undernutrition (stunting and wasting) in adolescents has detrimental effects, as it affects their ability to learn and work at maximal productivity. It affects their sexual maturation, increases the risk of poor obstetric outcomes for females and jeopardizes the healthy development of future children [10]. Obesity is a risk factor for a range of conditions including cardio-vascular disease, diabetes mellitus, arthritis and some cancers [16]. Concern about obesity is particularly important in adolescents because of their increased interest in physical appearance, self esteem and an associated poor self image.

The weight status of children and adolescents is often measured using Body Mass Index (BMI) and compared with reference standards. The BMI is an anthropometric index of weight and height that is defined as body weight in kilograms divided by height in meters squared [17]. BMI is the most widely used and simplest anthropometric index for assessing the weight status of children and adolescents since it can be used to identify those who may be overweight, at risk of being overweight, or underweight based on age and sex [18].

Few studies in Africa that used the WHO recommended references to assess the weight status of adolescents, documented the prevalence of undernutrition (BMI <5^th^ percentile of the WHO/NCHS reference) to be between 4–30% [11-13]. In South Asia, a high prevalence of about 50% was found among adolescents [14,19,20]. In Nigeria, there is scanty information on the weight status of adolescents and no available reference standard of their BMI exists. Port Harcourt, the oil city of Nigeria has a mixed population of residents ranging from high to low socioeconomic class. The town has experienced rapid population growth due to oil exploratory activities with overcrowding and springing up of many fast food outlets. The effects of these factors on the weight status of the adolescents have not been examined. This study therefore attempts to evaluate the weight status of adolescents in Port Harcourt using BMI, identify factors influencing it, with a view to developing and producing a reference standard of BMI among adolescents in our environment.

## Materials and methods

Over a 3 week period in April 2010, a cross-sectional descriptive study was carried out in Port Harcourt City, capital of Rivers State of Nigeria.

### Sample

A stratified multi staged sampling method was used to select the students for the study. A total of 8 schools (4 private, 4 public) composed of 4 co-educational, 2 all girls and 2 all boys were selected by simple random sampling. Nine hundred and sixty (960) Students aged between 10 and 19 years from the selected secondary schools were recruited into the study. Adolescents with chronic illnesses like heart diseases, asthma or disabilities like scoliosis and kyphosis were excluded from the study.

### Permission for the study

Permission for the study was obtained from the Research and Ethics Committee of the University of Port Harcourt Teaching Hospital and Post Primary School Education Board, while consent was obtained from individual school principals and parents/students.

### Questionnaire

Information on the questionnaire included the students personal data, parental occupation and level of education, medical history and average number of hours spent watching television per day. The nutritional history comprised of the number of meals consumed on an average day as well as a 24 hour dietary recall. The students were also asked the frequency of snack and beverage consumption on an average week. Examples of snacks specified included pastries, biscuits, as well as chocolates and sweets, while beverages included soft drinks, processed juices and energy drinks.

Socioeconomic stratification was done based on the classification described by Oyedeji [21]. Occupation and educational attainments of parents were used to determine the socioeconomic index scores of the subjects. Each student was assigned scores based on parents (father and mother’s) education and occupation. The scores were summed up and the mean (approximated to the nearest whole number) obtained. The mean score was used to assign the subject to one of the socioeconomic groups (I-V). The social classes of the subjects were further stratified into upper (social classes I and II), Middle (social class III) and lower (social classes IV and V).

Anthropometric measurements comprising of weight and height were measured on each subject and recorded on the questionnaire. BMI was calculated using the formula weight/height^2^ (kg/m^2^).

### Procedure for field work

Over a period of two days, five research assistants who were post internship doctors were trained by the investigators, who are Paediatricians. During the training, the investigators and research assistants practiced how to position the students to remove error of parallax and how to adjust the scale to zero before each weight measurements. They were also trained on how administer and fill the questionnaires. The questionnaires were pre-tested and validated one month to the time of the study.

On the first day of the study, the investigators and research assistants went to the selected schools to familiarize themselves with the school authorities and the students. During this period, a brief talk on nutrition, complications and prevention of malnutrition states was given to the teachers and students. The objective of the study was clearly explained to the students. Each student was given a consent form which he/she took home and brought back the next day. On subsequent days, the selected students were seated in the school hall, and the consent forms collected. One questionnaire per student was administered and filled by the investigators and assistants. Anthropometric measurements comprising of weight and height were measured for each student and recorded on the questionnaire. At the end of each study day, all completed questionnaires were retrieved and standardized by one of the investigators.

### Anthropometric measurements

Weight was measured using a well-calibrated, portable bathroom scale (Hana scale, model BR-9011). Students were weighed standing on the scale with their shoes off. The scales were checked before each measurement for zero adjustment and standardized according to WHO recommendations [22].

Height was measured using a portable stadiometer, which consisted of an anthropometer with a simple triangular headboard. In taking the height the students were made to stand straight with their shoes off and head held erect such that the external auditory meatus and the lower border of the eye were in one horizontal plane (Frankfurt plane). The buttocks, shoulder blades, and heels touched the scale with knees and legs together, and arms hanging naturally by the side. A movable triangular headboard was brought against the crown of the head and the height measurement read off at maximum inspiration to the nearest centimeter.

All measurements were taken twice by the one of the investigators and an assistant and the average taken. A third measurement was taken if the first two differed by > 0.5 kg in weight and 0.5 cm in height, to avoid inter-observer error. Only one of the investigator and an assistant did all the anthropometric measurements to avoid intra-observer error.

### Weight status reference standard

Body mass index was calculated using the formula weight/height^2^ (kg/m^2^). Those subjects whose BMI for age were < 5^th^ percentile of the National Centre for Health Statistics (NCHS) reference population were considered to be underweight, those whose BMI for age were between 5^th^ and 85^th^ were considered as having normal weight, ≥ 85^th^ but < 95^th^ percentile were considered to be at risk of being overweight. Those > 95^th^ percentile were said to be obese and those whose height for age is < 3^rd^ percentile were said to be stunted [23].

### Data analysis

Data was analysed using the Statistical Package for Social Sciences (SPSS) software version 14^85^ and Epi Info version 6.04. Analysis of variance was used to test statistical significance with respect to continuous variables while Chi-square was used for discreet variables. A probability value of less than 0.05 was considered statistically significant at 95% confidence interval.

## Results

### Age and gender distribution of study population

A total of 960 students were studied. The students’ age ranged from 10 to 19 years with a mean of 14.25 ±  2.19 years. There were 481 males (50.1%) and 479 females (49.9%) with M: F ratio of 1:1. The mean age of males was 14.49 ± 2.29 years, while that of females was 14.01 ± 2.05 years. The difference in age between sexes was not statistically significant except for those aged 18 and 19 years of age. Table 1 shows age and gender distribution of subjects.

**Table 1:** Distribution of subjects by age and gender

**Age (Years)**	**Males No. (%)**	**Females No. (%)**	**Total**	**χ**^**2**^	**P value**
10	15 (3.1)	25 (5.2)	40	2.65	0.10
11	32 (6.7)	27 (5.6)	59	0.43	0.51
12	61 (12.7)	71 (14.8)	132	0.93	0.33
13	60 (12.5)	71 (14.8)	131	1.12	0.29
14	80 (16.6)	81 (16.9)	161	0.01	0.90
15	74 (15.4)	92 (19.2)	166	2.45	0.12
16	54 (11.2)	56 (11.7)	110	0.05	0.82
17	50 (10.4)	35 (7.3)	85	2.04	0.09
18	35 (7.3)	15 (3.1)	50	0.35	0.00*
19	20 (4.2)	6 (1.3)	26	7.69	0.01*
**Total**	**481 (100)**	**479 (100)**	**960**		

### Stage of adolescence by gender

More than half (54.5%) of the subjects were in early adolescence, of these, 277 (53%) were females as shown in Table 2. There were 76 (7.9%) subjects in late adolescence, with a male preponderance of 72.4%. The gender difference was only statistically significant in late adolescence p = 0.000

**Table 2:** Stage of adolescence by gender

**Age Group(years)**	**Male (%)**	**Female (%)**	**Total**
Early 10–14	246 (47.0)	277 (53.0)	523 (100)
Mid 15–17	180 (49.9)	181 (50.1)	361 (100)
Late 18–19	55 (72.4)	21 (27.6)	76 (100)
**Total**	**481**	**479**	**960**

### Mean Body Mass Index (BMI) for age by gender

A steady increase in growth was reflected by the BMI which showed a gradual increase with age (Table 3) except at 11 years in males and 19 years in females. The mean BMI at 10 years for both sexes was 16.68 ± 2.34 kg/m^2^ and by 19 years it had risen to 21.89 ± 2.15 kg/m^2^. The overall mean BMI for females (20.01 ±3.50 kg/m^2^) was significantly higher than that of males (19.01 ±2.58 kg/m^2^), (p = 0.000).

**Table 3:** **Mean BMI (kg/m**^**2**^**) at various ages by gender**

**Age**	**Males**		**Females**		**P value**
**(Years)**	**No.**	**Mean ± SD**	**No.**	**Mean ± SD**	
10	15	17.25 ± 2.66	25	16.34 ± 2.11	0.20
11	32	16.20 ± 1.68	27	17.22 ± 3.60	0.70
12	61	17.38 ± 2.21	71	19.21 ± 3.09	0.00*
13	60	18.00 ± 2.41	71	19.84 ± 3.07	0.00*
14	80	19.06 ± 2.29	81	20.13 ± 2.93	0.01*
15	74	19.61 ± 1.99	92	20.34 ± 2.90	0.06
16	54	19.50 ± 1.78	56	21.38 ± 4.59	0.00*
17	50	20.72 ± 2.44	35	21.57 ± 3.05	0.15
18	35	20.82 ± 2.29	15	23.23 ± 3.20	0.00*
19	20	21.60 ± 2.15	6	22.85 ± 2.07	0.22
**Total**	**481**	**19.01 ± 2.58**	**479**	**20.01 ± 3.50**	0.00*

* = Significant

### Prevalence of malnutrition using BMI percentile by gender

Table 4 showed that 61 (6.4%) of the study population were underweight. Majority (85.3%) had normal weight, while the prevalence of obesity was 1.8%. According to gender, significantly more males (8.9%) were underweight compared to females 3.8% (p = 0.000). Females were significantly more overweight and obese than males (p < 0.05)

**Table 4:** Weight status by gender

**Weight status**	**Sex**		**Total**	**χ**^**2**^	**P value**
**(NCHS)**	**Males No. (%)**	**Females No. (%)**			
Normal	417 (86.7)	402 (83.9)	819 (85.3)	1.47	0.220
Underweight	43 (8.9)	18 (3.8)	61 (6.4)	10.83	0.000
Overweight	18 (3.7)	45 (9.4)	63 (6.3)	12.50	0.000
Obese	3 (0.6)	14 (2.9)	17 (1.8)	7.29	0.006
**Total**	**481 (100)**	**479 (100)**	**960 (100)**	**29.20**	**0.000**

### Prevalence of stunting

A total of 52 (5.4%) students were stunted (height-for-age < 3^rd^ percentile of NCHS reference standard). More males (7.9%) were stunted compared to females (2.9%). The observed difference was statistically significant (p = 0.000, *χ*^2^ = 11.61) as shown in Table 5.

**Table 5:** Height for age percentile according to gender

**Height for age**	**Male No %**	**Female No %**
Stunted	38 (7.9)	14 (2.9)
Normal	443 (92.1)	465 (97.1)
Total	481 (100)	479 (100)

### Prevalence of stunting according to stage of adolescence

Stunting occurred more in mid-adolescence than early or late adolescence in both sexes. In all stages of adolescence, males were more stunted than their female counterparts, except in mid-adolescence where females were more stunted. These differences were however not statistically significant (Table 6).

**Table 6:** Prevalence of stunting according to stage of adolescence by gender

**Period of adolescence**	**Gender**		**Total**	**χ**^**2**^	**P value**
	**Male No. (%)**	**Female No. (%)**			
Early	9 (23.7)	3 (21.4)	12	0.04	0.84
Mid	22 (57.9)	11 (78.6)	33	1.89	0.17
Late	7 (18.4)	0 (0.0)	7	1.61	0.20
**Total**	**38 (100)**	**14 (100)**	**52**		

### Effect of social characteristics on weight status

Factors which were commoner in overweight adolescents were high socioeconomic class, higher maternal education, spending > 3 hours a day watching television and frequent ingestion of snacks (Table 7).

**Table 7:** The relationship between certain social factors and television viewing on weight status

**Characteristic**	**Normal No %**	**Underweight No %**	**Overweight No %**	**Obese No %**	**Total**
**Social class**					
Upper	244 (84.4)	12 (4.1)	25 (8.7)	8 (2.8)	289 (100)
Middle	327 (86.7)	23 (6.1)	20 (5.3)	7 (1.9)	377 (100)
Lower	248 (84.4)	26 (8.8)	18 (6.1)	2 (0.7)	294 (100)
**Mother’s education**					
No education	47 (90.4)	4 (7.7)	1 (1.9)	0 (0.0)	52 (100)
Primary	139 (87.4)	10 (6.3)	9 (5.7)	1 (0.6)	159 (100)
Secondary	358 (86.1)	26 (6.3)	24 (5.8)	8 (1.9)	416 (100)
Technical/Commer	55 (85.9)	5 (7.8)	3 (4.7)	1 (1.6)	64 (100)
Higher/University	220 (81.8)	16 (5.9)	26 (9.7)	7 (2.6)	269 (100)
**Family size**					
≤5	198 (84.6)	19 (8.1)	13 (5.6)	4 (1.7)	234 (100)
6–10	563 (85.7)	36 (5.5)	45 (6.8)	13 (2.0)	657 (100)
11–15	58 (84.1)	6 (8.7)	5 (7.2)	0 (0.0)	69 (100)
**Hours spent watching TV**					
0–2	477 (86.1)	33 (6.0)	37 (6.7)	7 (1.3)	554 (100)
3–4	238 (85.0)	19 (6.8)	19 (6.8)	4 (1.4)	280 (100)
≥5	104 (82.5)	9 (7.1)	7 (5.6)	6 (4.8)	126 (100)
**Snack intake/week**					
Once	101 (87.1)	5 (4.3)	6 (5.2)	4 (3.4)	116 (100)
1–2	137 (87.3)	11 (7.0)	9 (5.7)	0 (0.0)	157 (100)
>3	199 (86.4)	13 (5.7)	13 (5.7)	5 (2.2)	230 (100)
Everyday	382 (83.5)	32 (7.0)	35 (7.7)	8 (1.8)	457 (100)
**Soft drink/week**					
Once	320 (84.2)	26 (6.8)	24 (6.3)	10 (2.6)	380 (100)
1–2 times	254 (87.0)	20 (6.8)	15 (5.1)	3 (1.0)	292 (100)
>3	161 (84.3)	11 (5.8)	16 (8.4)	3 (1.6)	191 (100)
Everyday	84 (86.6)	4 (4.1)	8 (8.2)	1 (1.0)	97 (100)

## Discussion

The mean BMI of females in this study was significantly higher than that of males from 11 years of age throughout adolescence. Similar trend was observed by Ijarotimi et al. [15], Ukegbu [24] and Mukhopadhyay et al. [14]. This is different from NHANES findings in which the BMI of males and females were almost identical. This difference in the BMI between sexes may be the result of increased fat mass in females in contrast to males who stabilize their fat mass and enlarge their fat free mass [13]. The fact that males are taller than females may also have contributed to their low BMI since height is a denominator in calculating BMI. Also decreased physical activity in females may result in storing of calories which contributes to their increased weight [25].

Eighty-five percent of the study population had normal weight. This is agreement with previous studies [24,26]. Majority of the normal weight subjects were males.

The prevalence of underweight in this study was 6.4%, which contrasts with findings from previous studies with underweight prevalence of 33.1% [26] in Philippines and 20% [27] in Nigeria. In the Philippine study [26], although the study population was similar to that of the present study, their sample size was much larger (6079) and therefore would be more representative of the total population. This could explain the disparity between this study and that reported in their study. The low prevalence in this study may probably be due to exclusion of adolescents with chronic illnesses. Although, Ukegbu et al. [24] studied adolescents in mid and late adolescence (15–18 years) who should have a low prevalence of underweight, the high prevalence obtained in their study may be because their study population consisted of boarding school students, compared to day students who are likely to have more access to nutritious and well balanced food.

The overall overweight prevalence of 6.3% was similar to that in the Philippine study of 7.3% [26]. Females were more overweight than their male counterparts. This however differed from Ukegbu’s [24] study where the prevalence of overweight was lower in females than in males. This difference cannot be readily explained as females are generally known to have higher subcutaneous fat and BMI than their male counterparts. Al-Saheed et al. [28], in Saudi Arabia reported a higher overweight prevalence of 20%. This may be due to their study group which included children 6–17 years of age. The preadolescents are known to have higher overweight rates [4] and coupled with higher socio-economic standards in their country [29], one is not surprised at the high prevalence of overweight in their study.

The prevalence of obesity (BMI equal or greater than the 95^th^ percentile for age and sex) in this study was 1.8%. This is in agreement with other studies by Alabi [27] in Port Harcourt and Izuora [30] in Lagos. Females were significantly more obese than males. The lower prevalence of obesity in males may be the result of higher degree of physical activity [25]. In Ukegbu’s study [24] no obese adolescents were found, this was probably due to the small sample size. This prevalence rate of 1.8% is much lower than results obtained in developed and more affluent industrialized countries like USA (15%), UK (20%), France (14%), Russia (6.7%), and China (3.6%) [31].

The extent of height deficit in relation to age may be regarded as a measure of the duration of malnutrition. Height is affected not only by chronic malnutrition but also by genetic and hormonal factors [32]. The low prevalence of stunting (5.4%) reported in this study was similar to that reported by Brabin et al. [33] in Port Harcourt in 1997 in a study of South-eastern Nigerian adolescent girls and de-Onis et al. [34] in Calcutta, India. Although they used less or equal to second centile for height-for-age of British Reference standard and –2SD Z-scores of NCHS reference as cut-off point, it however differed from other studies by Ukegbu et al. [24] who reported stunting rates in males and females with an overall prevalence of 62.5% in both sexes. The reason for this enormous difference is not clear. The essential differences in the study population in both studies are the age ranges of the subjects and their tribes being predominately Igbos and Ijaws in Ukegbu’s study [24] and the present study respectively. Further investigations need to be done to determine if the differences in age and tribe significantly affected the heights of the subjects. In the present study, subjects with chronic illnesses were excluded, as chronic illnesses usually account for most cases of stunting in our environment. Therefore the exclusion of subjects with chronic illnesses may be responsible for the low prevalence found in this study. Generally, males are more stunted than their female counterparts [24,26], this was similar to findings in this study.

Socioeconomic status (SES) affects access to culturally appropriate and affordable food, thus affecting the quality of diet. The prevalence of underweight in this study was higher in the lower SES as compared to the upper SES, where overweight and obesity was found to be higher in the higher SES. This is not surprising as there is growing evidence that perhaps due to decreased physical activities, sedentary lifestyle, altered eating patterns and increased fat content of the diet the prevalence of overweight/obesity is higher in the upper SES. The relationship between obesity and socioeconomic status varies across countries. The higher the socioeconomic class (SEC) the more the risk of obesity in Russia and China, while in USA, the lower the SEC the higher the risk of obesity [35]. In the USA, obesity is more prevalent among the lower SEC and this has been attributed to the theory that food deprivation or the fear of deprivation can lead to overeating when food is available [36]. Consumption of junk food has been associated with incidence of obesity.

This study revealed that subjects who ingested beverages everyday tended to be overweight. Although the authors did not come across similar studies, Dehghan et al. [31], reported that excessive beverage intake has been associated with epidemic of obesity and type II diabetes mellitus in children and adolescents. This may be explained by the fact that adolescents who ingest beverages daily tend to fill their stomachs with these carbonated drinks with high sugar and caloric content which promote weight gain.

The study also revealed that the adolescents who ingested snacks everyday were more underweight than those who took only once a week. This may also be explained by the fact that daily ingestion of these highly processed snacks with poor nutritional value will consequently cause reduction in appetite and consumption of nutritious foods provided at home.

Television viewing greater than 3hours per day was associated with increased prevalence of overweight and more than 5hours a day with more obese subjects. The risk associated with this behavior may operate through several mechanisms, including reduction of time spent in higher intensity activities, a lowering of metabolic rate and more frequent snacking [37]. It is known that fast foods are frequently advertised on television. Children and adolescents are often the targeted market, therefore it is not surprising that there is increased snacking while viewing television [31].

Another finding in this study was worsening of the nutritional status of subjects with increasing family size. Although this finding was not statistically significant, it is similar to findings from another study in children less than five years which showed an association between nutritional status and family size [38]. This is in line with the findings of other authors who found that subjects from small family sizes, higher socioeconomic class, with highly educated mothers tended to be more obese [31].

## Conclusion

The overall mean BMI for females was significantly higher than that of males while the males were significantly more stunted than females. Adolescents from upper social class, whose mother’s had higher education and spent more than 3hours watching television tended to be more overweight than the counterparts whose parents were from lower social class and spent less hours watching television.

Periodic weight assessment of adolescents should be carried out in schools and communities as part of school health programme. This is essential for early detection, planning and implementation of intervention programmes to reduce morbidity and mortality associated with under and overnutrition. Also, health education to promote healthy eating behaviors, regular physical exercise and regulated television viewing should be inculcated into the school curriculum. This would contribute to controlling overweight and obesity.

## Competing interests

The authors declare that they have no competing interest.

## Authors’ contributions

AFA conceived of the idea for the study, designed the questionnaire, collected and analyzed the data, OP wrote the manuscript, IA and NA both revised the manuscript and made significant intellectual contributions. All the authors read and approved the final manuscript.
